# Research on Anomaly Identification and Screening and Metallogenic Prediction Based on Semisupervised Neural Network

**DOI:** 10.1155/2022/8745036

**Published:** 2022-07-21

**Authors:** Rongqing Zhang, Zhenzhu Xi

**Affiliations:** ^1^Key Laboratory of Metallogenic Prediction of Nonferrous Metals and Geological Environment Monitoring (Central South University), Ministry of Education, Lushan Road, Changsha 410083, China; ^2^Key Laboratory of Non-Ferrous Resources and Geological Hazard Detection, Central South University, Lushan Road, Changsha 410083, China; ^3^School of Geosciences and Info-Physics, Central South University, South Lushan Road, Changsha 410083, China

## Abstract

This paper firstly introduces the background of the research on neural network and anomaly identification screening and mineralization prediction under semisupervised learning, then introduces supervised learning, semisupervised learning, unsupervised learning, and reinforcement learning, analyzes and compares their advantages and disadvantages, and concludes that unsupervised learning is the best way to process the data. In the research method, this paper classifies the obtained geochemical data by using semisupervised learning and then trains the obtained samples using the convolutional neural network model to obtain the mineralization prediction model and check its correctness, which finally provides the direction for the subsequent mineralization prediction research.

## 1. Research Background

China is a vast country with extremely rich resources of various kinds. There are two kinds of resources used by human beings in today's world, one is renewable resources and the other is nonrenewable resources. Mineral resources, as a limited resource, are nonrenewable resources, compared with renewable resources such as rare metals, nonferrous metals, alloys, and rubber. Although China is a large energy country, but in the late Qing Dynasty after the crazy plunder and exploitation of imperialism, nowadays the per capita possession of mineral resources is extremely small, and the special geological environment of mineral resources, the problem of unreasonable resource structure division has led to the development of China's mineral business is not smooth. At the same time, according to President Xi's concept of “green water and green mountains are the silver mountain of gold,” and with the in-depth development of the theory of mineralization prediction, we should survey and protect the limited mineral resources to ensure that our mineral resources can be effectively developed and utilized, without damaging the environment. In this paper, the anomaly identification screening and prediction study of the mining area is completed based on the semisupervised learning approach of neural network [1].

The next section describes the background of the development of neural networks and anomaly screening and prediction of mineralization based on mineral resources in a semisupervised learning approach, respectively.

### 1.1. Neural Networks under Semisupervised Learning Approach

As more and more mineral resources are developed, the theory of mineralization prediction in China has also been developed and the introduction of neural networks under deep learning in artificial intelligence into geology has become a major trend and research hotspot [2]. In order to make a better prediction of mining area, we first understand the background of the development of neural network under semisupervised learning approach [3].

The term “semisupervised neural network” refers firstly to the neural network model based on deep learning techniques and secondly to the semisupervised learning approach used in the training of the neural network model [4].

Early neural networks are called SNNs, which are shallow neural networks. DNNs are called deep neural networks, which are much more layered and deeper than SNNs, but both SNNs and DNNs are artificial neural networks, i.e., ANNs.

The development of neural networks can be divided into three phases, with the first phase starting in the 1940s and ending in the 1970s. The year 1943 was the seminal year when Warren McCulloch and Walter Pitts proposed a mathematical model of formal neurons and expressed the concept of what an artificial neural network is in their article “A logical calculus of the ideas immanent in nervous activity” [5]. The formulation of this mathematical model and the definition of the concept directly determined the birth of neural networks. However, the initial mathematical model of formal neuron was not perfect, and the most essential defect was that there was no suitable algorithm to adjust the weights of the neuron model due to the limitation of the development of technology, so it did not receive much attention when it was first proposed [6]. In 1958, Rosenblatt et al. proposed the “perceptron” based on the error learning algorithm, which means that the neural network model can be trained to adjust the weights, and the output of the perceptron is continuously adjusted by the error to make the actual output gradually approximating the predicted output, which is equivalent to connecting the weights of the neural network [7]. From the introduction of the mathematical model of formal neural networks (M-P model) to the emergence of “perceptrons,” the first wave of research based on neural networks was launched. However, in the subsequent research on perceptrons, it was found that there was a fatal flaw in perceptrons, i.e., they could only deal with linearly divisible problems and could only solve single-layer linear problems, but could not do anything for linearly indivisible problems because they could not use multi-layer networks.

Thus, the development of neural networks ushered in the second phase, whose second phase spanned a decade. In the early 1980s, Hopfield proposed a new network, the HNN network (Hopfield neural network), based on the research boom of neural networks [8]. In order to solve the shortcomings of the perceptron in the linear indistinguishability problem, by the end of 1980s, Rumelhart (Rumelhart) and others proposed a new algorithm-BP algorithm (error backpropagating algorithm) in the article “Learning representations by backpropagating errors.” This algorithm is essentially a *δ*-algorithm, which is based on the principle of solving the linear indistinguishability of the perceptron by setting up multiple perceptual layers (implicit layers) and propagating them either forward or backward through the process. Due to the emergence of BP algorithm, the development of neural networks has seen a second boom. In this context, algorithms based on neural network models are fruitful, for example, in 1989, based on the application of recognizing handwritten digits, Yann Lecun and other scholars implemented a CNN network with seven layers, namely LeNet-5. In this application, the accuracy rate of recognizing handwritten digits could reach 98% [9]. During this period, the industrial revolution was also in full swing, and thanks to the development of technology, a large number of researchers conducted further research on the HNN network proposed by Hopfield, creating a new boom. However, the boom was limited again with the rise of other machine learning algorithms, including SVM (support vector machine), whose advantages were much higher than those of the neural networks, and thus, the development of neural networks fell into a slump [10].

After decades of downturn, in the early-mid 2010s, research scholars such as Jeff Hinton proposed to start modeling neural networks layer by layer based on RBM (i.e., restricted Boltzmann machine), using the training method of modeling successive layers of neural networks to extract high-dimensional features from the training set data, and based on this, the concept of deep learning and deep networks, i.e., deep belief networks-multilayered ANNs (artificial neural networks) was developed. This approach was used by many researchers and scholars to model different neural networks due to its ability to greatly improve the generalization of models, and neural networks thus led to the third climax. In the following decade or so, neural networks have remained hot and are widely used in image recognition, pattern recognition, speech recognition, machine translation, and other fields. At present, there are many deep belief network models that have been proposed, such as convolutional neural network CNN, graph neural network GNN, etc. [11].

For example, Deng Hao et al. used deep learning techniques in their paper “Three-Dimensional Mineralization Prediction and Quantitative Analysis of Tectonic Control Factors in Jiaojia Gold Belt Based on Attentional Convolutional Neural Network” to establish mineralization control indicators and a three-dimensional geological model by introducing a convolutional neural network model, including the addition of CBAM attentional mechanism module, to obtain the initial mineralization control indicators after obtaining useful mineralization information features from the initial mineralization control indicators, a simple nonlinear relationship between the fracture surface and mineralization localization was established, and the conclusion of the study proved that new mineralization enrichment zones may exist in the deep part of the connection area between Jiaojia and Qujia Kancha [12]. In order to break through the difficulty of finding cryptomagnetism, Miao Guowen et al. carried out a study of mineralization prediction based on BP artificial neural network and practiced in the Cocosili Lake area in Qinghai. Nine units were selected for prediction and a BP-ANN cryptomagnetism prediction model was constructed, and their results showed that the Cocosili Lake in Qinghai does contain cryptomagnetism. This shows that neural networks bring great convenience in mineralization prediction, and also bring hope for the further development of mineralization prediction theory [13].

### 1.2. Anomaly Identification Screening and Mineralization Prediction Theory

Anomaly identification and screening refers to the screening of chemical prospect anomalies, which was first proposed in 1993 when researchers discussed the evaluation and screening methods of regional chemical prospect anomalies in response to the shortage of arranging anomaly examination, mainly using the comprehensive information scoring method and the expert prediction evaluation method. Subsequently, in order to further explore the mineral search potential of the shallow coverage area, Dai Yonggang made his elemental anomaly map by clustering the elements obtained from the analysis after processing the anomaly rejection, etc., of the data in the Kansai area, and after circling more anomalies, finally compared the circled anomalies with the known deposit types using gray correlation analysis, so as to screen out the favorable mineral anomalies [14]. After years of development, anomaly screening and identification have been carried out in related areas. For example, Yang Limin and other researchers selected and evaluated geochemical anomalies in Ulan Duran area of Qinghai Province, applied systematic kernel and kernel degree theory, fully analyzed and studied the technical methods, achieved excellent application results, and further studied the anomalies, which provided further anomaly examination and exploration of mining areas. Scientific basis [15].

Ore deposit formation prediction refers to some theoretical analysis on prediction, such as the prediction of various resources in the block, the prediction analysis of mineralization type, origin, etc., From a historical point of view, the development process of mineral formation prediction has gone through three main stages. In the second stage, in the 1970s and 1980s, due to the development of computer technology and multivariate statistical methods, some researchers innovatively applied them to mineralization prediction, thus opening a new chapter in mineralization prediction. At the same time, expert systems were also introduced into mineralization prediction models during this period, such as the medium- and large-scale mineral deposit statistical prediction expert system (MILASP) established by the research group led by academician Dapeng Zhao in the paper “Implementation of an Expert System for Model Unit Selection Based on Rule-Based Knowledge Representation.” The third stage is after 1980s, due to the development of industry, the supply of mineral resources exceeds the demand and there is a trend of shortage, thus mineralization prediction has been greatly developed in the first stage, and GIS technology has been applied to mineralization prediction model, for example, by the construction of mineralization in the Lancang River basin in Yunnan, mainly Chi Du Shun, GIS technology, i.e., GIS, was applied to establish the mineral resource potential, the spatial analysis model of mineral resource potential evaluation, and the quantitative analysis of mineralization intensity and breadth, etc. [16].

In the mineral prediction for the 21st century, the development of mineralization theory is constantly being broken, but the mineral resources are also shrinking, so it seems urgent to use new ways to find mineral resources. In this paper, we will identify anomalies and predict mineralization by using neural network with semisupervised learning method to screen the resources in the mining area of Bajiazi area in Zalantun City, Inner Mongolia, and build a mineralization prediction model by using its geochemical data.

## 2. Geological Setting

In this paper, we investigate the geological environment and formation process of the mining area in Bajiazi, Zalantun City, Inner Mongolia Province, and combine the neural network with semisupervised learning method for anomaly identification and mineralization prediction model.

First of all, it is known from the literature that the Late Paleozoic Upper Carboniferous-Lower Permian Gegen Ovoo Group, Mesozoic Upper Jurassic Manitou Group, and Quaternary alluvium are mainly exposed in the area [17]. The volcanic rocks are mainly the Late Paleozoic Upper Carboniferous-Lower Permian Gegen Ovoo Group, Mesozoic Upper Jurassic Manitou Group, and Quaternary alluvium [18]; the intrusive rocks are mainly P1*γδ* (Early Permian light gray medium fine-grained granodiorite), K1*γo* (Early Cretaceous fine-grained plagioclase granite), and T3*ηγ* (Late Triassic medium fine-grained diorite granite). The main vein rocks are amphibolite (*δμ*) and orthogeneous porphyry (*ξπ*).

## 3. Learning Mode of Neural Networks

The composition of neural network is similar to the human brain activity, both are simple mathematical models composed of many neural units through certain connections compared to the complex brain activity, and they are used to simulate the process of human brain activity. The learning mode of neural networks can be divided into supervised learning, semisupervised learning, reinforcement learning, and unsupervised learning.

With the in-depth study of mineral prediction theory, the data about mineral resources are becoming more and more complicated. Neural network is proposed according to human learning ability and brain activity, and the combination of neural network and mineral prediction can process the relevant information well and train the relevant data with neural network model to improve the correctness of mineral prediction model.

### 3.1. Supervised Learning

The flow chart of supervised learning is shown in Figure 1. Supervised learning is a way of learning a neural network model by first learning the training data with labels to obtain a new model, and then using this model to predict the output of the new sample data [19]. In this case, the word “supervised” means that the training samples, i.e., the expected output (label) of the input data, are already known. The process of using the new model to make predictions on the new sample data is called mapping, and this mapping relationship is represented by a model, which is equivalent to a function in a mathematical equation [20].

In terms of mathematical space, the sample input is equivalent to the set of input space and the output is the set of output space, and the model represents the mapping relationship from the set of input space to the set of output space [21]. Determining the spatial set relationship means that the learning range is determined. Finding the best mapping relationship within that learning range is the essence of supervised learning.

The framework of supervised learning process can be broadly divided into two parts: learning and prediction.

In the learning process, it is actually the process of determining the model, as shown in Figure 2. In this process, feature vectors are first extracted from the data in the training set, which can be textual information, photos, etc., [22]. The feature vector extraction process is then completed by extracting the desired features from the data. Next, some machine learning algorithm is used to iteratively train the input data with labeled information and the feature information in the training set to finally form a new model suitable for conducting experiments. Then, the feature vectors of the new training set are obtained by extracting the feature information of the new training set using the same feature extraction method. Finally, by inputting the feature vectors of the new training set into the new model, the prediction of the new samples is completed in the new model, and the predicted classification results of the new samples are finally obtained [23].

### 3.2. Reinforcement Learning

Reinforcement learning also belongs to machine learning. The purpose of reinforcement is to reinforce the learning of knowledge with the fundamental aim of developing an intelligent body or system [24]. Its intelligences or systems are able to improve the performance of their learning experience by interacting with the environment, and in reinforcement learning, a reward mechanism is usually included. A reward mechanism means that if an intelligence or system completes a certain type of learning and gets the correct answer, it is given a reward in order to motivate it to keep reinforcing the learning.

The main components of reinforcement learning are the environment and the intelligence, with secondary factors such as state, reward, and strategy [25]. The intelligence, the subject of reinforcement learning, is the equivalent of a learner or decision maker. The environment, on the other hand, consists mainly of the set of states, which refers to everything outside the reinforcement learning system or the intelligent body. The state in reinforcement learning represents the data in the environment, and the state set is all possible states in the environment [26]. In reinforcement learning, an intelligence learns by reinforcement in the environment, and after learning, it can acquire the corresponding experience, i.e., it can perform certain actions, and the set of these actions is called the action set; the action set is the set of all behaviors that the intelligence can perform [27]. After acquiring an action or behavior, it is judged whether it can be rewarded according to a given judgment criterion. Therefore, in the feedback of reinforcement learning, the feedback is not the label of the data or other data that the system model considers useful as in supervised learning, but the result of whether the reward function is satisfied with the action or behavior of the intelligence [28]. If the reward function is satisfied with the intelligence's performance, it will judge to give a reward, otherwise it will be judged as unsatisfactory and continue the reinforcement learning after giving a punishment. It can be seen that agents (intelligences) can achieve reinforcement learning by interacting with the environment and maximize this reward through exploratory trial and error or careful planning [29].

Representative algorithms for reinforcement learning are the SARSA (state-action-reward-state-action) algorithm and Q-learning algorithm based on tableaux; the DQN algorithm based on neural networks and the policy-gradient algorithm based on policy gradients. In the SARSA algorithm, due to the exploratory nature in reinforcement learning, it is necessary to use the e-greedy algorithm when executing the next step thus achieving the updated Q value, i.e., the next action needs to be made before the Q value can be updated again; in the Q-learning algorithm, the biggest difference with the SARSA algorithm is the different way of updating the Q table, using the way of “off-policy,” this way does not need to know the next action, instead it assumes that the next work step has then taken the maximum value of Q. However, this traditional table-based approach requires a large amount of storage when encountering large-scale learning tasks, which leads to the problem of inefficient execution. In response to the shortcomings of SARSA (state-action-reward-state-action) algorithm and Q-learning algorithm, deep Q-learning algorithm is proposed. The basic idea of DQN algorithm is to adopt the neural network approach to approximate instead of Q forms, and its innovation lies in experience playback and Q target fixation.

In contrast to supervised learning, the most important feature of reinforcement learning is the reward mechanism. While supervised learning is a class of machine learning based on the label of known training data, reinforcement learning is a feedback to the environment so that the benefit of the intelligence in action can be maximized. Although reinforcement learning does not require a priori knowledge of the known training set, it requires feedback on the actions in the environment at each step due to its reward mechanism, which is judged by the reward function. Since the criterion of judgment is the reward function, it means that the feedback is quantifiable and reinforcement learning is an act of giving feedback to continuously adjust the learning object of the model.

### 3.3. Semisupervised Learning

In the process of training a model using supervised learning, a new model is obtained by training a training set with known prediction results using machine learning algorithms using existing prior knowledge. This type of learning requires experience before it can be performed, i.e., if the data without labels have to be manually labeled, it greatly wastes human and material resources and greatly limits the scope of its application. In reinforcement learning, the interaction between the environment and the intelligence is achieved through the feedback mechanism of the reward function, so that there is no need to obtain the label of the training set data in advance, which can reduce the processing of the data and thus make the algorithm procedure relatively simple, but the mechanism of reinforcement learning makes it less likely to achieve more complex learning behaviors. Semisupervised learning, on the other hand, is a class of machine learning approaches that are intermediate between supervised and unsupervised learning [30]. Its workflow is shown in Figure 3.

Semisupervised learning is a class of machine learning that takes advantage of existing labeled data. Semisupervised learning is a class of machine learning that uses existing labeled data to train on unlabeled data to obtain more labeled data.

### 3.4. Unsupervised Learning

The fundamental difference between unsupervised learning and supervised learning, or semisupervised learning is whether the input data are labeled or not; if the input data are labeled, the learning method is called supervised learning; if some of the input data are labeled and some are not, the learning method is called semisupervised learning; if all the input data are unlabeled, the learning method is called unsupervised learning, i.e., clustering [31].

Unsupervised learning is characterized by the fact that the data passed to the algorithm is abundant in the internal structure in the neural network, but there are fewer words used for reward or training. The essence of an unsupervised learning algorithm can be understood as the data itself, rather than as a specific task. Due to its learning style, unsupervised learning is often used in data mining to find patterns in large unlabeled data and use the sample patterns to analyze the training or test set. Although unsupervised learning can be used for data mining and data analysis, the unsupervised learning approach does not require labeling of the data, so the neural network models trained under the unsupervised learning approach may not capture the expected criteria in mind, and the accuracy of data processing using the unsupervised learning approach is more than a dozen percentage points lower than that of supervised or semisupervised learning.

### 3.5. Summary

To address the problems of high reliance on a priori knowledge in supervised learning, difficulty in handling high complexity in reinforcement learning, and low correctness in unsupervised learning for processing data, this paper addresses the problem of reducing the reliance on a priori knowledge in training models by combining neural network models with semisupervised learning methods. In addition, since the neural network model can adaptively adjust its internal structure based on the training sample data set itself, combining with the semisupervised learning approach can also enhance its adaptive adjustment capability. Therefore, the training model used in this paper for anomaly screening and mineralization prediction in the Bajiazi area of Zalantun City, Inner Mongolia Province, is a neural network-based mineralization prediction model with semisupervised learning approach [32].

## 4. Research Methodology

In this paper, we firstly use the neural network model with semisupervised learning to classify the geochemical data to provide a data base for mineralization prediction; secondly, we identify and screen the anomalies in the mining area with this learning method, and then build a mineralization prediction model for the classified geochemical data and test the accuracy of the training under the neural network.

### 4.1. Neural Network Model under Semisupervised Learning Approach

#### 4.1.1. Neurons

The neural network model under semisupervised learning approach is firstly introduced in this paper. The basic unit of a neural network is a neuron, which can also be referred to as a node. The neuron structure is shown in the figure below.

From Figure 4, it can be seen that the neuron model is composed of multiple inputs and one output. In the process of input to output, it goes through the summation and nonlinear function. Before the summation, the input to summation process is adjusted by the weights, and each input corresponds to a different weight. The arrows in the diagram indicate the “connections.” The nonlinear function refers to the activation function, where different activation functions and weights correspond to different outputs in the neuron.

#### 4.1.2. Selection of Activation Functions

The common activation functions include sigmoid and ReLU. Nair and Hinton applied the rectified linear unit (ReLU) to the neural network in 2010, which is known from Figure 5 and equation (1): the ReLU function is actually a segmented linear function. Observing its function image can be obtained that the function can return all values less than 0 to 0, while the values greater than 0 remain unchanged, i.e., one-sided suppression. This one-sided inhibition method sparsely activates the neurons in the neural network, giving the neurons the property of sparse activation. In particular, in deep neural network models (e.g., CNN), the activation rate of ReLU neurons is theoretically reduced to half of the Nth power when N layers are added to the model. The sparse model implemented by the ReLU activation function can better mine relevant features and adapt them to the training data, reducing the occurrence of overfitting.

(1) $$\begin{array}{c} f\left(z\right)=\max\left(\text{0,}z\right). \end{array}$$

In this paper, the activation function used is the ReLU function in order to improve the robustness and generalization ability of the model. The ReLU function is chosen because the linear composite function has the problem of limited fitting ability, so the activation function is introduced to transform the simple mapping of the model into a nonlinear mapping, which helps to improve the expressiveness of the model. At the same time, the ReLU function is not as susceptible as other complex activation functions, and the function model is also simple thus simplifying the computational process. At the same time, the decentralization of activity reduces the cost and the overall computational complexity of the entire neural network.

#### 4.1.3. Convolutional Neural Networks

Unlike conventional neural networks, which do not have a convolutional layer, convolutional neural networks have this layer and the neurons in each layer are arranged in 3 dimensions: width, height, and depth. The convolutional neural network is shown in the following figure.

As shown in Figure 6, the first light blue rectangle on the left represents the input layer, and the dark blue rectangle connected with the light blue on the left is the neuron after convolution and pooling, which can also be regarded as the activation value, followed by the convolutional pooling layer and the fully connected layer, and the fully connected layer followed by the output layer. The convolutional layer, the fully connected layer, and the pooling layer form the hidden layer of the multi-layer perceptron.

Next, each layer is constructed in this neural network model.

Convolutional layers: each convolutional layer of a convolutional neural network consists of several convolutional units, and the parameters of each convolutional unit are optimized by a back propagation algorithm. The purpose of the convolutional operation is to extract various features of the input vector. The first convolutional layer may extract only some low-level features, such as edges, lines, corner points, etc., More layers of the convolutional network can iteratively extract more complex features from lower-level features. In this case, the convolutional layer performs feature extraction on simple cells in the local sensory field through weight sharing and local connectivity. Different features of the input signal are extracted by multiple convolution operations, one feature per convolution kernel, so that *n* features can be extracted by *n* convolution kernels.

Pooling layer: usually after the convolution layer, a feature of large dimension is taken, that feature is cut into several regions, a maximum or mean value is taken, and a new feature of small dimension is taken. The role of pooling layer is to reduce the parameter variables of the network model by gradually reducing the spatial size of the data volume, which not only can effectively know the generation of overfitting phenomenon, but also can reduce the consumption of computational resources.

Fully connected layer: after the convolution and pooling layers, each node is connected to the fully connected layer by a “join.” This means that all local features are combined with global features, thus turning the features of the former into all features of the latter. Adding a fully connected layer will help improve the network performance of the convolutional neural network for calculating the final score of each class.

#### 4.1.4. The Loss Function

In this paper, we use cross entropy as the loss function in our study, which is used to find the gap between the predicted value and the target. First of all, entropy is the knowledge in Shannon's information theory, to understand the principle of cross entropy one must first understand what is the amount of information. The amount of information, i.e., the amount of useful information obtained from an event. The amount of information is related to probability, generally, the greater the probability of something happening, the greater the amount of information contained in that event. Entropy, on the other hand, is the mathematical expectation of the amount of information. In machine learning, the probability *P* is often the true distribution of the sample, not the ideal distribution, and the predictive model should also contain the predictive distribution *Q*. If there is a relative information increment of *P* for *Q*, the KL scatter can be used to describe the difference between these two distributions. If *Q* is repeatedly trained to describe the probability distribution *P* perfectly, then the “information increment” is not needed and the training model is excellent. The KL dispersion is calculated as follows, where *n* is the probability of all events.

(2) $$\begin{array}{c} D_{KL}\left(p\|q\right)=\prod_{i=1}^{n}p\left(xi\right)\mathrm{lo}g_{10}\frac{p\left(x_{i}\right)}{q\left(x_{i}\right)}. \end{array}$$

Equation (3) can be obtained by deforming equation (2).

(3) $$\begin{array}{c} D_{KL}\left(p\|q\right)=\prod_{i=1}^{n}p\left(xi\right)\mathrm{lo}g_{10}\left(q\left(x_{i}\right)\right)-\left[\prod_{i=1}^{n}p\left(xi\right)\mathrm{lo}g_{10}\left(q\left(x_{i}\right)\right)\right], \end{array}$$

where the cross entropy is the first part of the −∏_*i*=1_^*n*^*p*(*xi*)log_10_(*q*(*x*_*i*_)) equation, which is generally equated to H(p,q). Since the gap between labels and predictions needs to be evaluated in this study, it is appropriate to use the KL scatter, but again, since the first part of the KL scatter is constant, it is only necessary to note the change in the cross entropy. So, in this study, the loss function directly uses the cross entropy for the evaluation model.

#### 4.1.5. Data Processing

The data in this study were obtained from the geochemical data of the Bajiazi mining area, and the elemental content of the samples of the geological entities was examined by laboratory assay means, and the obtained chemical data were manually labeled in order to perform semisupervised classification of the resulting data sources using semisupervised learning. This study focuses on the prediction and analysis of Pb elements in the region.

### 4.2. Anomaly Identification Screening of Neural Networks in a Semisupervised Learning Approach

The researchers identified an integrated anomaly through soil measurements. The anomaly was located in the southwest of the Kansa area with an overall circular distribution. The Ag-Pb-Zn-Cd-Cu-As anomaly is large and moderate in intensity and scale due to its dominance. The anomalies of each element are highly similar and have linear local characteristics with the north-east and north-west-west distribution. Second, on small scales, Mo, Au, Sb, Bi, W, and Sn elements anomalies are highly consistent across elements.

It shows that the soil contains various elements and mineral veins. Symbols 13 and 14 represent abnormal contour and abnormal high value points, respectively, and symbol 15 represents element abnormality. The comprehensive analysis shows that the mineralization and alteration state of Bajiazi mine is good, the Ag, Pb, Zn, and other multi-element anomalies match well, and it has the characteristics of low-resistance and high-polarization anomalies. The comprehensive geological and chemical exploration characteristics can well predict the mineralization, which provides an effective basis for future mineral exploration.

### 4.3. Application of Neural Network for Mineralization Prediction under Semisupervised Learning Method

In this paper, the Pb elements in the geochemical data of the Bajiazi area are used as the input vector of the convolutional neural network, and the SoftMax layer is used as the output layer to output the probability of each type. The loss function is cross entropy. The detection results of the final mineralization prediction model in this paper are shown in the following Figure 7.

As can be seen from Figure 7, the accuracy of the metallogenic prediction model reaches a more stable state at 600 iterations with an accuracy rate of about 85%, which proves the feasibility and effectiveness of the model.

## 5. Conclusion and Outlook

In this study, a neural network mineralization prediction model based on the neural network under semisupervised learning approach was developed in the context of introducing the neural network model under semisupervised learning approach, and the geological analysis of the mining area in the Bajiazi area of Zalantun City, Inner Mongolia Province, and its geochemical data were used as the research object. In the description of the model, the basic unit of the neural network model, neuron, is firstly described, followed by the selection of the appropriate activation function for the model, RELU activation function, and finally the training of the convolutional neural network model to establish the mineralization prediction The model was tested for its correctness, and the experimental results showed that the correctness rate was about 85%. However, the experimental study still has some shortcomings, such as the need for manual labeling of geochemical data processing, which can be improved in the future.

### 5.1. Conclusion

In this study, in the context of introducing the neural network model under semisupervised learning approach, the geological analysis of the mining area in the Bajiazi area of Zalantun City, Inner Mongolia Province, and its geochemical data were used as the research object to establish the neural network mineralization prediction model based on the semisupervised learning approach. In the elaboration of the model, the basic unit of the neural network model, neuron, is firstly elaborated, followed by the selection of the appropriate activation function for the model, RELU activation function, and finally by training the convolutional neural network model to establish the mineralization prediction The model was tested for its correctness, and the experimental results showed that the correctness rate was about 85%. However, the experimental study still has some shortcomings, such as the need for manual annotation of geochemical data processing, which can be improved in the future.

## Figures and Tables

**Figure 1:** Flowchart of supervised learning.

**Figure 2:** Flowchart of supervised learning applied to classification prediction.

**Figure 3:** Semisupervised learning on classifier.

**Figure 4:** Basic neuron model.

**Figure 5:** Image of the function of ReLU function.

**Figure 6:** Basic structure of a convolutional neural network.

**Figure 7:** Accuracy of the training of the convolutional neural network mineralization prediction model for Pb elements in the Bajiazi mining area in Inner Mongolia.

## Data Availability

The labeled dataset used to support the findings of this study are available from the corresponding author upon request.
